The article "Sepsis-induced elevation in plasma serotonin facilitates endothelial hyperpermeability" was retracted in 2019. Reasons: errors in the images; original data or images not available.

# Sepsis-induced elevation in plasma serotonin facilitates endothelial hyperpermeability

**DOI:** 10.1038/srep22747

**Published:** 2016-03-09

**Authors:** Yicong Li, Coedy Hadden, Anthonya Cooper, Asli Ahmed, Hong Wu, Vladimir V. Lupashin, Philip R. Mayeux, Fusun Kilic

**Affiliations:** 1 Departments of Biochemistry and Molecular Biology, University of Arkansas for Medical Sciences, Little Rock, Arkansas, US; 2 Departments of Physiology University of Arkansas for Medical Sciences, Little Rock, Arkansas, US; 3 Pharmacology and Toxicology, University of Arkansas for Medical Sciences, Little Rock, Arkansas, US

## Abstract

Hyperpermeability of the endothelial barrier and resulting microvascular leakage are a hallmark of sepsis. Our studies describe the mechanism by which serotonin (5-HT) regulates the microvascular permeability during sepsis. The plasma 5-HT levels are significantly elevated in mice made septic by cecal ligation and puncture (CLP). 5-HT-induced permeability of endothelial cells was associated with the phosphorylation of p21 activating kinase (PAK1), PAK1-dependent phosphorylation of vimentin (P-vimentin) filaments, and a strong association between P-vimentin and ve-cadherin. These findings were in good agreement with the findings with the endothelial cells incubated in serum from CLP mice. *In vivo*, reducing the 5-HT uptake rates with the 5-HT transporter (SERT) inhibitor, paroxetine blocked renal microvascular leakage and the decline in microvascular perfusion. Importantly, mice that lack SERT showed significantly less microvascular dysfunction after CLP. Based on these data, we propose that the increased endothelial 5-HT uptake together with 5-HT signaling disrupts the endothelial barrier function in sepsis. Therefore, regulating intracellular 5-HT levels in endothelial cells represents a novel approach in improving sepsis-associated microvascular dysfunction and leakage. These new findings advance our understanding of the mechanisms underlying cellular responses to intracellular/extracellular 5-HT ratio in sepsis and refine current views of these signaling processes during sepsis.

Sepsis is an extremely complex medical condition characterized by a severe systemic inflammatory response caused by a microbial infection. Patients with severe sepsis have a poor prognosis with mortality rates of 40–60% when one or more organs are affected (reviewed in *1, 2*)^1^,^2^. Microvascular dysfunction is a hallmark of sepsis and is believed to contribute significantly to patient mortality. The endothelial cell lining of the microvasculature is the first line of defense against organ injury during sepsis. As such, it is susceptible to injury from microbial virulence factors, proinflammatory mediators released from activated blood cells, and oxidative stress^3^. It is generally agreed that endothelial dysfunction promotes the neutrophil adhesion and infiltration into tissues, coagulation abnormalities, microvascular leakage, and hypoperfusion associated with sepsis-induced multiorgan failure.

The article "Sepsis-induced elevation in plasma serotonin facilitates endothelial hyperpermeability" was retracted in 2019. Reasons: errors in the images; original data or images not available.

Recent publications underscore the complex role platelets play in the inflammatory response, hemostasis, host response, and microvascular permeability during sepsis^3^,^4^,^5^,^6^,^7^. Platelets become activated during sepsis and release a variety of mediators that affect coagulation and endothelial function^8^. One such mediator is serotonin (5-hydroxytryptamine, 5-HT), which is stored in dense granules of platelets and released into the plasma during platelet activation. 5-HT is a multifunctional signaling molecule and can mediate a number of cellular functions including regulation of cytoskeletal dynamics associated with barrier function^9^,^10^,^11^,^12^,^13^. Therefore, the concentration of 5-HT in the blood is tightly regulated by a specific 5-HT transporter (SERT) expressed on the surface of the platelet and endothelial cell, which removes 5-HT from the blood and increases intracellular 5-HT levels. Although, 5-HT signaling can increase permeability of the endothelial barrier^12^,^13^, its role in microvascular leakage during sepsis has not been fully investigated.

To examine the functional role of 5-HT in microvascular failure during sepsis, we used a clinically relevant murine model of polymicrobial sepsis induced by cecal ligation and puncture (CLP) and evaluated the renal microcirculation by intravital microscopy and measured renal microvascular leakage. Initial studies examined the mechanism by which 5-HT affects the endothelial barrier and were performed in an *in vitro* model of murine renal endothelial cells exposed to septic serum or 5-HT and evaluated endothelial barrier function. Data demonstrate that plasma levels of 5-HT are elevated during sepsis, which triggers increased uptake of 5-HT by endothelial SERT. Earlier studies connected plasma 5-HT and activation of p21 activating kinase (PAK1), which phosphorylates vimentin on residue Ser56^14^,^15^,^16^. Following phosphorylation, vimentin undergo spatial reorganization, which affects the proteins in association with P-vimentin such as ve-cadherin. Our data provide evidence that this reorganization weakens the endothelial cell permeability barrier. Importantly, the pharmacological inhibitor of SERT, paroxetine, reduced renal microvascular leakage and improved renal microvascular perfusion. Based on these data, we propose that controlling the rates of 5-HT uptake may represent a novel approach to alleviating sepsis-associated microvascular dysfunction and leakage by taking advantage of the endogenous SERT uptake mechanism already in place.

The article "Sepsis-induced elevation in plasma serotonin facilitates endothelial hyperpermeability" was retracted in 2019. Reasons: errors in the images; original data or images not available.

## Results

### Platelets are activated rapidly during sepsis in the mouse

Platelets isolated from mice at 4 h following induction of sepsis by CLP displayed a significant increase in the aggregatory response to collagen compared to platelets isolated from SHAM mice (Fig. 1A) as noted in previous studies^3^,^8^.

Platelets are the major storage for 5-HT in blood, which is released during platelet activation^17^. Therefore, 5-HT levels in the plasma of CLP or SHAM mice blood samples were determined using a competitive ELISA technique (Fig. 1B). Plasma 5-HT concentration was 4.38 ± 0.16 nM in the blood samples of SHAM mice but 13.16 ± 0.83 nM in the blood samples of 4 h post CLP mice. Platelets isolated at 4 h post CLP displayed a significant (1.37-fold) increase in SERT activity compared to platelets isolated from SHAM mice (Fig. 1C). These data suggest that both 5-HT uptake rates of platelets and plasma 5-HT levels increase rapidly in septic mice.

### Septic serum alters endothelial cell function

We previously showed that 4-h CLP serum induces oxidative stress in mouse renal epithelial cells and mimics renal epithelial injury observed *in vivo* in the CLP model^18^,^19^. Next, the impact of CLP on endothelial 5-HT uptake was investigated in mouse endothelial cells (2H11) cultured in serum samples prepared from 4 h post CLP or SHAM mice. The 5-HT uptake rates of endothelial cells cultured in 5% CLP was 1.57-fold higher (P < 0.01) compared to endothelial cells cultured in SHAM serum for 45 min (Fig. 2A).

5-HT is known to increase the permeability of blood vessels^12^,^13^. Furthermore, 5-HT signaling regulates the formation of P-vimentin via activation of PAK and disassembly and spatial reorientation of vimentin filaments in smooth muscle and CHO cells^14^,^15^,^16^. Here, the mechanism in which 5-HT signaling modulates the association between ve-cadherin and P-vimentin was evaluated in endothelial cells. The endogenous expression of three proteins, vimentin, P-vimentin and ve-cadherin were detected in endothelial cells cultured in SHAM or CLP serum at 55-, 55- and 132-kDa bands as shown in Fig. 2B. After detecting the endogenous expression of vimentin, P-vimentin and ve-cadherin in endothelial cells by Western blot (WB) analysis, we tested an association between vimentin or P-vimentin with ve-cadherin in the lysates of the endothelial cells grown in SHAM or CLP mouse serum for 24 h by immunoprecipitated (IP) assay. IP was performed with monoclonal ve-cadherin Ab and the ve-cadherin immune precipitates were resolved by SDS-PAGE and then subjected to WB with polyclonal Ab against vimentin or P-vimentin (pS56-Ab). Our data revealed that ve-cadherin was co-isolated with vimentin and P-vimentin (Fig. 2C). However, in endothelial cells exposed to SHAM serum the level of P-vimentin isolated from ve-cadherin complex was 1.3-fold less than in the endothelial cells exposed to CLP serum. The vimentin Ab can recognize vimentin and P-vimentin however, our custom made P-vimentin Ab, pS56 only recognizes P-vimentin^16^. Control experiments performed in the absence of ve-cadherin Ab failed to isolate vimentin- or P-vimentin-cadherin complex. Thus, the level of P-vimentin found on ve-cadherin Ab appeared much higher than the level of vimentin in endothelial cells cultured in CLP serum.

The article "Sepsis-induced elevation in plasma serotonin facilitates endothelial hyperpermeability" was retracted in 2019. Reasons: errors in the images; original data or images not available.

Elevated 5-HT activates PAK to phosphorylate vimentin on serine 56^14^,^15^,^16^. Based on these data we hypothesize that an association between P-vimentin and ve-cadherin may play a major role in the cellular and molecular mechanisms of the endothelial dysfunction during sepsis. This hypothesis was explored in 5-HT pretreated endothelial cells.

### Characterization of 5-HT pretreated endothelial cells

Our earlier studies established that the 5-HT uptake rates of platelets show a relationship to plasma 5-HT concentrations^20^. Specifically, the 5-HT uptake rates of platelets initially rise as plasma 5-HT levels are increased, but then fall below normal as the plasma 5-HT level continues to rise. To examine whether this phenomena also occurs in endothelial cells, we exposed 2H11 endothelial cells for 45 min with various concentrations of 5-HT (0 to 300 μM) then measured 5-HT uptake rates. 5-HT level in SHAM plasma was determined ~ 5 nM and in CLP it was ~ 13 nM. However, the translation of these *in vivo* findings to an *in vitro* experimental condition required 5-HT treatment several-fold greater in order to induce a similar effect. This could be a result of *in vivo* conditions not replicated in culture experiments. For example, the effects of 5-HT may be enhanced when endothelial cells are lining the vascular wall and exposed to flow-induced shear stress. As observed in platelets^20^ endothelial cells also displayed a transient increase in 5-HT uptake rates with 20 μM 5-HT pretreatment (Fig. 3A). The 5-HT uptake rate of platelets from CLP mice was 1.37-fold higher than the platelets of SHAM mice (Fig. 1B). Similarly, the endothelial cells pretreated with 20 μM 5-HT showed 1.6-fold higher 5-HT uptake rates compared to the untreated endothelial cells which is similar to the level found in the plasma of septic mice.

To assess whether the increase in 5-HT uptake rate might be due to an increase in the surface expression of SERT, 2H11 cells were treated with 5-HT at concentrations of 0, 20 μM or 100 μM for 45 min then subjected to surface biotinylation followed by western blot analysis for SERT. Data in Fig. 3B showed that 20 μM 5-HT increased SERT expression on the plasma membrane by 1.56-fold compared to the untreated control group of cells, which corresponded to reduction in intracellular SERT expression by 1.66-fold. In contrast, a higher concentration of 100 μM 5-HT did not change the level of SERT on the surface significantly or at the intracellular compartments (Fig. 3B).

The article "Sepsis-induced elevation in plasma serotonin facilitates endothelial hyperpermeability" was retracted in 2019. Reasons: errors in the images; original data or images not available.

We next evaluated the effects of 20 μM 5-HT treatment on P-vimentin levels in 2H11 cells by immunofluorescence (IF) and WB analysis (Fig. 4A and B, respectively). 5-HT treatment caused a switch from vimentin to P-vimentin via changing the organization of this intermediate filament. In control cells the vimentin (green) was easily recognized with its bridging capacity between the cells, but P-vimentin appeared rarely (red). However, 5-HT pretreatment of endothelial cells elevated the level of P-vimentin significantly, which mostly appeared around the cellular membrane (Fig. 4A). The WB analysis of endothelial cells demonstrated the expression of P-vimentin in 5-HT treated group although residual levels of P-vimentin was found in control cells indicating that there are other factors involved in the P-vimentin formation beside 5-HT (Fig. 4B). Both approaches indicated that 20 μM 5-HT increased the phosphorylation of vimentin.

### 5-HT and the phosphorylation of vimentin

To investigate the mechanism by which 5-HT signaling modulates phosphorylation of vimentin, we first treated platelets from wild-type (WT) and SERT^−/−^ mice with 20 μM 5-HT 45 min at room temperature then analyzed the expression of P-vimentin (Fig. 4C). P-vimentin was only increased in 5-HT pretreated platelets of WT mice suggesting 5-HT modulates the phosphorylation of vimentin. Importantly, SERT^−/−^ mice could not phosphorylate vimentin in the presence of 5-HT, indicating that phosphorylation of vimentin requires SERT and an elevation in intracellular 5-HT concentration.

To explore whether this novel mechanism of 5-HT-mediated vimentin phosphorylation occurs in endothelial cells, 2H11 cell were incubated with 20 μM 5-HT for 24 h in the presence of the calcium-dependent transglutaminase (TGase) inhibitor cystamine (Cys)^21^ or the SERT inhibitor paroxetine (PAR)^20^. Endothelial cells, stimulated with 20 μM 5-HT showed a 5.5-fold elevation in the level of P-vimentin. This elevation was reduced in the presence of Cys or PAR (Fig. 5A). Based on these findings we hypothesized that 5-HT activates PAK1 to its phosphor-PAK1 form. Therefore, next we tested this hypothesis by analyzing the endothelial cells pretreated with 5-HT and Cys in WB using phospho-PAK1 (P-PAK1)-Ab. Endothelial cells were first incubated with TGase or a specific PAK1 inhibitor, PAK1-18 (EMD-Millipore, Billerica MA). At the end of 20 min, 20 μM 5-HT added to the incubation media and the incubation continued for an additional 30 min. The cells were then lysed and a portion of the cell lysate was analyzed by WB (Fig. 5B). In co-IP assays, vimentin-ve-cadherin association was tested in the remaining cell lysate (Fig. 5C). The phosphorylation of p-PAK1 was elevated 5.5 fold with 5-HT pretreatment. This effect was blocked by pretreatment with Cyst to block 5-HT transport and by PAK1 inhibition with PAK18 (Fig. 5B). Cyst and PAK18 also blocked cadherin-P-vimentin association (Fig. 5C). Taken together, the data suggest that 5-HT activates PAK, which in turn activates P-vimentin.

The article "Sepsis-induced elevation in plasma serotonin facilitates endothelial hyperpermeability" was retracted in 2019. Reasons: errors in the images; original data or images not available.

### Serotonylation of Rac

TGase transamidates 5-HT on the GTP-GDP hydrolysis domain of Rac which keeps this small GTPase in its active form, Rac-GTP^22^,^23^,^24^. This process was first described as serotonylation of small GTPases by Diego Walther *et al.*^25^. Endothelial cells were incubated with ^3^H-5HT for 1 hr, followed by a radioimmuno precipitation (RIP) on Rac coated protein A beads. Samples from: (i) whole platelet lysates to measure the total radioactive material in platelet; (ii) the eluent of protein A beads coated with Rac-Ab to measure the level of radioactive material associated with the Rac-Ab; and (iii) depleted platelet lysate to measure the amount of radioactive material left after Rac-Ab pull down from the whole platelet lysate, were all normalized for protein concentration. Then, samples from each group were measured in the scintillation counter (Fig. 6). The Rac-Ab bound proteins were resolved by SDS-PAGE and subjected to fluorography. One major band was observed at 25 kD as shown in Fig. 6. We were able to observe the serotonylation Rac in the endothelial cells pretreated with 20 μM 5-HT. Levels of Rac, SERT and actin were unchanged in endothelial cell lysates.

We next hypothesized that the initial uptake of 5-HT by endothelial SERT, and prior to the down-regulation of SERT as an end-effect of serotonylation, is the critical event establishing the dysfunctional endothelia from 5-HT-treatment. To test this hypothesis, we pretreated endothelial cells with a well-characterized inhibitor of SERT, PAR or TGase, Cyst prior to 5-HT treatment. In the presence of PAR or Cyst, 5-HT treatment of endothelial cells did not produce ^3^H-5HT labeled Rac suggesting the involvement of TGase and SERT in serotonylation of Rac. The levels of 5-HT in the cell cytoplasm versus extracellular surface is an important factor in transformation of Rac to GTP form.

The article "Sepsis-induced elevation in plasma serotonin facilitates endothelial hyperpermeability" was retracted in 2019. Reasons: errors in the images; original data or images not available.

### 5-HT and endothelial dysfunction

The level of 5-HT in the plasma can regulate the integrity of the endothelial cell barrier^12^,^13^. To evaluate this, murine endothelial cells (2H11 cell line) were grown to confluency on Transwell-COL plates then incubated for 45 min with 0, 20 μM or 100 μM 5-HT. At the end of the incubation period, FITC-dextran (40 kDa) was added to the monolayer and its appearance in the lower compartment was measured after 30 min. 5-HT treatment with 20 μM but not 100 μM increased permeability (Fig. 7). This response was similar to what was observed with SERT activity in endothelial cells (Fig. 3A). These finding suggested that leakage might be dependent on SERT activity. To address this we evaluated the effect of PAR on 5-HT-induced leakage and found that leakage was completely blocked by PAR (Fig. 7), implicating a key role for SERT in regulating the endothelial permeability barrier in response to 5-HT.

### Role of SERT in renal microvascular dysfunction following CLP

One of the earliest events in the kidney following CLP is an increase in renal capillary leakage^26^. At 4 h post CLP, renal microvascular permeability as measured by Evans Blue dye accumulation in the kidney was significantly increased compared to SHAM (Fig. 8A). To investigate the role of SERT, mice were treated with PAR (4 mg/kg, ip) or vehicle (10% DMSO in saline) at the time of CLP. PAR prevented the increase in renal microvascular leakage (Fig. 8A). At 6 h post CLP renal cortical capillary perfusion was assessed using intravital video microscopy (IVVM). IVVM allows measurements of capillary perfusion in real time in live anesthetized animals^26^. CLP produced a significant decline in the percentage of vessels with continuous flow and an increase in vessels with no flow (Fig. 8B). To investigate the role of SERT on perfusion, wild-type mice treated with PAR and SERT^−/−^ mice were subjected to CLP and perfusion was measured at 6 h. Capillary perfusion was improved in mice treated with PAR (4 mg/kg, ip, at the time of CLP) and in SERT^−/−^ mice compared to wild-type (WT) mice (Fig. 8B). Representative still images from the videos are presented in Fig. 8C with arrows indicating renal cortical peritubular capillaries with no flow.

These data suggest that 5-HT uptake by SERT is critically linked to both decreased microvascular perfusion and increased microvascular leakage during sepsis. Moreover, the findings indicate that targeting SERT can provide functional protection of the microvasculature during sepsis.

The article "Sepsis-induced elevation in plasma serotonin facilitates endothelial hyperpermeability" was retracted in 2019. Reasons: errors in the images; original data or images not available.

## Discussion

Microvascular failure, including hypoperfusion and loss of the endothelial permeability barrier, is a hallmark of sepsis in humans and linked to increased mortality^27^,^28^,^29^. In the CLP murine model of sepsis, renal microvascular failure is one of the earliest events to occur in the kidney and is linked to acute kidney injury^26^,^30^,^31^.

The endothelial permeability barrier is maintained through interactions between complex sets of proteins that comprise tight junctions, adherens junctions, and gap junctions. Adherens junctions form pericellular zipperlike structures along the cell border through their transmembrane homophilic adhesion^32^. Endothelial adherens junctions contain vascular endothelial (ve)-cadherin as the major structural protein that mediates homophilic binding and adhesion of adjacent cells in a Ca^2−^-dependent manner. ve-Cadherin is required for the proper assembly of adherens junctions and development of normal endothelial barrier function^33^. We recently reported in the CLP model that the renal microvascular permeability barrier could be stabilized and even repaired by the sphingosine-1-phosphate receptor 1 agonist SEW2871^31^ or the phosphodiesterase 4 inhibitor rolipram^30^. In the present study we sought to address the mechanism in which 5-HT plays a role in de-stabilization of the endothelial permeability barrier during sepsis.

Endothelial cell activation during sepsis contributes to the activation of platelets, which release numerous mediators that affect coagulation and are believed to directly or indirectly affect the endothelial permeability barrier^34^. One such mediator is 5-HT, which can also be released from mast cells, the endothelium, and serotoninergic vascular nerves. 5-HT has been reported to increase the permeability of the endothelial cells in blood–brain barrier through a calcium-dependent signaling pathway^23^,^35^,^36^. This led us to examine the possible role of 5-HT in microvascular dysfunction during sepsis. At 4 h after induction of sepsis by CLP, platelets became hyperreactive as has been suggested to occur in humans with sepsis. Plasma levels of 5-HT were also significantly elevated in septic mice. This unique finding led us to examine the impact of 5-HT on endothelial cells.

The 5-HT uptake capacity of the cells depends on the number of SERT molecules on the plasma membrane. Earlier studies established that surface SERT expression in endogenous and heterologous expression systems shows a transient elevation with 5-HT at 20 μM concentrations. Specifically, plasma membrane SERT levels and 5-HT uptake by SERT initially rise as plasma 5-HT levels are increased, but then fall below normal as the plasma 5-HT level continues to rise. In *in vivo* and *in vitro* studies a dynamic relationship between the elevated extracellular/intracellular 5-HT ratios is associated with the intracellular trafficking and the loss of surface SERT^16^,^17^,^20^,^22^.

The article "Sepsis-induced elevation in plasma serotonin facilitates endothelial hyperpermeability" was retracted in 2019. Reasons: errors in the images; original data or images not available.

In a series of experiments in endothelial cells we found that 5HT-stimulation of cells activates p21 activating kinase (PAK), which in turn phosphorylates vimentin on the serine residue at position 56^14^,^15^,^16^. The effects of 5-HT on P-PAK formation were evaluated further to determine if it is direct or via an intracellular factor. Our earlier studies demonstrated that 5-HT signaling via IP3 signaling pathway elevates the intracellular Ca level^37^. This activates Ca-dependent enzyme transglutaminase (TGase)^22^,^24^. Endothelial cells pretreated with a TGase blocker, cystamine^21^ reduced phosphorylation of vimentin on Ser56 and the association P-vimentin-cadherin. These data suggest that 5-HT signaling on P-PAK formation is dependent on TGase activity. Seperately P-Pak formation is also related with the intracellular 5-HT in which PAR inhibited 5-HT uptake and P-PAK formation. Earlier, we showed that 5-HT activates TGase and transamidate intracellular 5-HT on small GTPases^24^. In endothelial cells, we propose that 5-HT signaling activates TGase to serotonylate Rac to active form Rac-GTP. Once Rac is serotonylated and becomes Rac-GTP, PAK1 becomes activated^37^ and active PAK1 phosphorylates vimentin.

Intermediate filaments are a major cytoskeletal component in endothelial cells^38^, but their role in endothelial permeability regulation is the least well understood. However, phosphorylation of vimentin occurred following stimulation of endothelial cells with agonists known to induce change in cell shape, 5-HT, thrombin, or phorbol esters^39^, implying that vimentin could influence endothelial barrier by an unknown mechanism. Biochemical studies have shown an association between vimentin and ve-cadherin^39^,^40^. Based on the reported studies and our data we hypothesize that an association between P-vimentin and ve-cadherin plays a major role in the cellular and molecular mechanisms of the endothelial dysfunction during sepsis. More specifically, an increased 5-HT signaling activate PAK1 and leads to the phosphorylation of vimentin continuously. This induces changes in the organization of vimentin-associated proteins and alters the barrier ability of endothelial cells. This feature of vimentin was observed in epithelial to mesenchymal transition^41^ also in the formation of lamellipodia^42^.

While platelets are recognized as modulators of vascular permeability^43^,^44^,^45^, the role 5-HT and its signaling pathways have not been well studied during sepsis. Our *in vitro* and *in vivo* studies suggest a new signaling pathway initiated during sepsis, which causes microvascular leakage (Fig. 9). This pathway is initiated by release of 5-HT from platelets and is dependent on SERT activity. The link between increased uptake of 5-HT by the endothelium and increased permeability is the activation of PAK1 and subsequent phosphorylation of vimentin and its increased association with ve-cadherin. The functional relevance of this new pathway was demonstrated in SERT^−/−^ mice, which displayed improved renal microvascular perfusion compared to wild-type mice following induction of sepsis by CLP. Moreover, pharmacological inhibition of SERT with paroxetine reduced microvascular leakage and also improved perfusion.

The article "Sepsis-induced elevation in plasma serotonin facilitates endothelial hyperpermeability" was retracted in 2019. Reasons: errors in the images; original data or images not available.

These findings are significant because septic patients still experience unacceptably high morbidity and mortality even when receiving guideline-approved goal-directed supportive therapy. SERT and 5-HT signaling should be considered as new targets for therapy development.

## Methods

### Animals

Adult male mice 36–40 weeks of age were used in these studies. C57BL/6J wild-type mice (WT) were purchased from Harlan (Indianapolis, IN) and SERT^−/−^ mice on a C57BL6 genetic background^46^ were purchased from The Jackson Laboratory (Bar Harbor, Maine). All animals were housed and euthanized in accordance with the National Institutes of Health Guide for the Care and Use of Laboratory Animals and with approval of the University of Arkansas for Medical Sciences Institutional Animal Care and Use Committee.

### Induction of sepsis by CLP

Polymicrobial sepsis was induced by CLP as described previously^26^. At the time of surgery, the mice were anesthetized using isoflurane inhalation. After laparotomy, a 4-0 silk ligature was placed 1.5 cm from the cecal tip. The cecum was punctured twice with a 21-G needle and gently squeezed to express approximately a 1-mm column of fecal material. In sham-operated mice, the cecum was located but neither ligated nor punctured. The abdominal incision was closed in two layers with 4-0 silk sutures. After surgery, 1 ml of prewarmed normal saline was given intraperitoneally. Mice were placed in individual cages and set on a warming pad.

### Renal microvascular permeability

Renal microvascular permeability was measured as described previously^31^. At 30 minutes before euthanizing, Evans blue dye (1% in 0.9% saline) was injected at 2 ml/kg via the tail vein. At euthanized, mice were perfused with 30 ml phosphate-buffered saline through the left ventricle until all blood was eliminated. The right kidney was weighed, homogenized in 1 ml formamide, and then incubated at 55 °C for 18 hours. The homogenate was then centrifuged at 12,000 x g for 30 minutes and the supernatant was collected. Evans blue dye was quantified in the supernatant by measuring absorbance at 620 nm and correcting for turbidity at 740 nm as described by Moitra *et al.*^47^. Concentrations of Evans blue dye were determined from a standard curve and expressed as μg/mg wet weight of the right kidney.

The article "Sepsis-induced elevation in plasma serotonin facilitates endothelial hyperpermeability" was retracted in 2019. Reasons: errors in the images; original data or images not available.

### Renal microvascular perfusion

Intravital video microscopy (IVVM) was performed as described previously^26^,^30^. Briefly, following anesthesia with isoflurane, FITC-labeled dextran (2 μmol/kg in 3 ml/kg normal saline) was administered via the penile vein to visualize the capillary vascular space. After 10 minutes, the left kidney was exposed by a flank incision and positioned on a glass stage above an inverted Zeiss Axiovert 200M fluorescent microscope equipped with an Axiocam HSm camera (Zeiss, Germany). Videos of 10 seconds (approximately 30 frames/second) at 200X magnification were acquired from five randomly selected, non-overlapping fields of view. Body temperature was maintained at 35°–37 °C with a warming lamp. Approximately 150 capillaries were randomly selected and analyzed from these fields of view from the kidney of each animal. Capillaries were categorized as “continuous” if red blood cell movement was uninterrupted; “intermittent” if red blood cell movement stopped or reversed; or “no flow” if no red blood cell movement was observed. Data were expressed as the percentage of vessels in each of the three categories.

### Quantitative measurement of 5HT levels by ELISA

The 5-HT levels in plasma which were prepared from the blood samples of each animal model was measured by competitive enzyme-linked immunosorbent assay (ELISA) technique by following the manufacturer’s instructions (IBL Immuno-Biological Laboratories, Hamburg, Germany) as described previously^20^,^22^.

### Stirred platelet aggregation

Blood samples were collected from the retro-orbital plexus using a glass capillary tube containing 3.8% sodium citrate solution. Platelet rich plasma (PRP) was prepared from whole blood^20^. Platelet counts were determined using a Hemavet 950 (Drew Scientific, Waterbury, CT) and adjusted to 300,000/μL with. Aggregation was initiated in PRP using collagen (3 μg/ml) and monitored by light transmittance using a platelet aggregometer (Chrono-log Corp., Havertown, PA)^20^,^22^.

### 5-HT uptake assay

Mouse endothelial cells (2H11 cells) were seeded 36–48 h in a Poly-D-lysine coated 24-well plate prior to initiating the transport assay. Uptake assays were performed by incubation of cells (2 × 10^5^ cells /assay) in 20.5 nM [1,2-^3^H (N)]-5-HT (14.6 nM final concentration; specific activity) 3400 cpm/pmol (Perkin Elmer Life Science) in PBS/CM (phosphate buffered saline 0.1 mM CaCl_2_ and 1 mM MgCl_2_) The intact cells were washed quickly with ice-cold PBS to stop the activity, harvested in 2% sodium dodecyl sulfate (SDS) in PBS, transferred to scintillation vials containing 5 ml scintillation cocktail, and the radioactivity was determined in a Beckman Scintillation Counter. An equal number of cells per cell line was confirmed by cell counting with a hemocytometer (Hausser Scientific, Horsham PA), and a group of cells were treated with a high-affinity cocaine analog, 0.1 μM 2β-carbomethoxy-3-tropane (β-CIT) to monitor 5-HT influx the background (β-CIT was provided by the Chemical Synthesis Service, National Institute of Mental Health)^20^,^22^.

The article "Sepsis-induced elevation in plasma serotonin facilitates endothelial hyperpermeability" was retracted in 2019. Reasons: errors in the images; original data or images not available.

### Western blotting (WB) analysis and quantitation of protein expression

Cells were lysed and solubilized in PBS containing 0.44% SDS, 1 mM phenylmethylsulfonyl fluoride (PMSF), and protease inhibitor mixture (PIM) which contained 5 mg/ml pepstatin, 5 mg/ml leupeptin, and 5 mg/ml aprotinin. Samples were analyzed by SDS-PAGE and transferred to nitrocellulose. Blots were incubated with primary Ab, rinsed, and then with horseradish peroxidase (HRP)-conjugated secondary Abs. The signals were visualized using the enhanced chemiluminescence (ECL) detection system. The polyclonal SERT Ab was generated by Proteintech Group, Inc. (Chicago, IL) on a peptide corresponding to the last 26 amino acids of the C terminus (positions 586–630) of SERT. Anti-SERT (diluted 1:500) gave one major band at 90 kD in endothelial cells. Signals were quantitated with a VersaDoc 1000 analysis system^22^. For determination of vimentin phosphorylation, membranes were probed with P-vimentin Ab which was generated by 21st Century Biochemicals, Inc. (Marlboro, MA) as described below.

### Anti-P-vimentin Ab (pS56-Ab)

Tang and co-workers^14^,^15^ raised an Ab for vimentin phosphorylated on serine 56. Using their approach as a guide, 21st Century Biochemicals, Inc. (Marlboro MA) synthesized a phosphopeptide against the sequence Ser-Leu-Tyr-Ala-Ser-phosphoSer56-Pro-Gly-Gly-Ala-Tyr-Cys and generated a site-specific polyclonal Ab for Ser-56 (anti-phosphovimentin (Ser-56) Ab). The affinity purified phosphovimentin Ab was first tested in endothelial cell lysate and mouse platelet and the findings were confirmed by using monoclonal vimentin- (cat # 904501, Biolegend in San Diego, CA) or polyclonal vimentin-Ab (cat. # sc-5565 Santa Cruz Dallas TX) which recognizes phosphorylated or unphosphorylated forms of vimentin. Our preliminary findings confirmed that P-vimentin (Ser-56) Ab can only recognize the P-vimentin phosphorylated on Ser56, as reported^16^.

The article "Sepsis-induced elevation in plasma serotonin facilitates endothelial hyperpermeability" was retracted in 2019. Reasons: errors in the images; original data or images not available.

### Cell surface biotinylation

Cell surface expression of SERT was detected after biotinylation with membrane-impermeant NHS-SS-biotin as described previously^16^,^20^,^22^,^24^. Briefly, upon the biotinylation reaction, the cells were treated with 100 mM glycine to quench unreacted NHS-SS-biotin and lysed in TBS containing 1% SDS, 1% TX100, and PIM/PMSF. The biotinylated proteins were recovered with an excess of streptavidin-agarose beads during overnight incubation. Biotinylated proteins were eluted in WB sample buffer, resolved by SDS-PAGE and transferred to nitrocellulose, and were detected as described^24^.

### Immunoprecipitation (IP)

Binding of ve-cadehrin to vimentin or P-vimentin was assayed in endothelial cells cultured in CLP or SHAM serum for 24 hrs or pretreated with 5-HT at indicated concentrations for 45 min at room temperature (RT). The cells were lysed in IP buffer (55 mM triethylamine [pH 7.5], 111 mM NaCl, 2.2 mM EDTA, and 0.44% SDS + 1% Triton X-100, 1 mM PMSF, PIM) and precleared by incubation with nonimmune rabbit serum and protein A for 1 hr and then centrifuged as described previously^16^,^20^,^22^,^24^. The precleared lysate was combined with an equal volume of a 1:1 slurry of protein A Sepharose beads and mixed overnight at 4^0^ C with a monoclonal ve-cadherin-Ab (Santa Cruz Dallas TX). Samples were separated on an SDS-PAGE and analyzed by WB with polyclonal anti-vimentin (Santa Cruz, Dallas TX) or P-vimentin (21st Century Biochemicals, Inc. Marlboro MA). The signals were developed with the ECL detection system.

For RIP, endothelial cells were treated with 20 μM cold and [^3^H]-5HT (100 μCi/ml) in PBS/CM at RT. After 1 hr, the cells were washed quickly with ice cold PBS and harvested, and Rac was IP using monoclonal Rac-Ab as described^22^. Immune precipitates were eluted from the beads by incubation in SDS sample buffer, analyzed by 12.5% SDS-PAGE, and visualized by fluorography.

### Immunofluorescence microscopy

Cells were plated on glass coverslips one day before 5-HT treatment. Cells were fixed and processed as described previously^48^. Fixed cell were incubated with anti-vimentin monoclonal Ab (cat # 904501, Biolegend in San Diego, CA) and S56 Abs followed by goat-anti-chicken-DyLight488 (Thermo Scientific, Rockford, IL) and goat-anti-rabbit-Alexa 555 (Molecular Probes). Cells were imaged with the 63X oil 1.4 NA objective of a LSM510 Zeiss Laser inverted microscope outfitted with confocal optics. Image acquisition was controlled with LSM510 software (Release Version 4.0 SP1).

The article "Sepsis-induced elevation in plasma serotonin facilitates endothelial hyperpermeability" was retracted in 2019. Reasons: errors in the images; original data or images not available.

### Macromolecular permeability assay

Mouse endothelial cells (2H11 cells) (0.125 × 10^6^ cells/well) were seeded on collagen G-coated 12-well Transwell^®^ plate inserts (pore size 0.4 μm, polyester membrane; Corning, New York, USA) and cultured for 48 h. FITC-dextran (40 kDa; 1 mg/ml; Sigma-Aldrich) was given to the upper compartment at t = 0 min. Cells were treated as indicated. Samples were taken from the lower compartment at t = 0/5/10/15/30 min. The fluorescence increase (ex 485/em 535) of the samples was detected with a fluorescence plate reader (SpectraFluor Plus, Tecan Deutschland GmbH). The mean fluorescence of untreated cells at t = 30 was set as 100%. The data are expressed as the percent increase of fluorescence versus the control.

### Data analysis

The *in vitro* data are presented as mean ± SD and the *in vivo* data are expressed as mean ± SEM. The Student’s t-test was used when two groups were compared, and a one-way analysis of variance followed by the Newman-Keuls post-hoc test was used when three or more groups were compared. Statistical significance was considered at P < 0.05.

## Additional Information

**How to cite this article**: Li, Y. *et al.* Sepsis-induced elevation in plasma serotonin facilitates endothelial hyperpermeability. *Sci. Rep.* **6**, 22747; doi: 10.1038/srep22747 (2016).

## Figures and Tables

**Figure 1:** (**A**) Platelet aggregation ratio. The elevated plasma 5-HT is associated with the increased aggregation rates of platelets. These were determined in the platelets (300,000 platelets/assay) of CLP and SHAM mice blood samples. The aggregation response to 3 μg/ml collagen was significantly (1.4-fold) higher in platelets from CLP mice compared to SHAM mice. Aggregation rates determined in three separate experiments (n = 4 each assay; *p *<* *0.001). (**B**) Characterization of 5-HT concentration in CLP- and SHAM mice blood plasma. 5-HT concentrations in blood plasma were measured by a competitive ELISA technique (4.38 ± 0.16 nM for SHAM (n = 4) and 13.16 ± 0.83 nM for CLP animals (n = 6)) as described previously^20^. Four hours post CLP application increased the plasma 5-HT concentration by 3–fold. (**C**) The 5-HT uptake rates of platelets isolated from CLP and SHAM mice blood samples. Plasma 5-HT level is regulated by SERT, a single gene product. Elevated plasma 5-HT was associated with a 1.37-fold increase in 5-HT uptake rates of platelets of CLP compared to the ones of SHAM mice. The rate of uptake is expressed as the mean ± SD of triplicate determinations from three independent experiments. *P* *<* *0.001 (compared with CLP *versus* SHAM uptake rates, respectively).

The article "Sepsis-induced elevation in plasma serotonin facilitates endothelial hyperpermeability" was retracted in 2019. Reasons: errors in the images; original data or images not available.

**Figure 2:** Endothelial cells incubated in CLP serum. (**A**) 5-HT uptake rates. Elevated plasma 5-HT was associated with a 1.57-fold higher 5-HT uptake rates of endothelial cells (2 × 10^5^ cells/assay) cultured in CLP compared to the ones incubated in SHAM serum. All assays were performed in triplicate. The rate of uptake is expressed as the mean ± SD of triplicate determinations from three independent experiments. *P* *<* *0.001(compared with cells cultured in CLP *versus* SHAM serum samples, respectively). (**B**) WB analysis of endothelial cells cultured in CLP or SHAM serum for P-vimentin and ve-cadherin. The endogenous expressions of vimentin, P-vimentin and ve-cadherin were identified with WB analysis of endothelial cells (2 × 10^5^ cells/assay) cultured in SHAM or CLP serum. No significant differences were detected in the total expression of vimentin and ve-cadherin between in endothelial cells treated with SHAM or CLP serum. (**C**) co-IP for endothelial cells cultured in CLP vs SHAM serum. Endothelial cells cultured in serum prepared from the blood samples of SHAM (S) or CLP mice. Next day the cell lysates were incubated with ve-cadherin monoclonal Ab coated protein A sepharose beads. The immunoprecipitates were subjected to WB analysis with vimentin or P-vimentin polyclonal Abs. The level of P-vimentin on ve-cadherin Ab was found elevated in cells cultured in CLP serum; however, no differences were found in the level of vimentin.

**Figure 3:** Endothelial cells pretreated with 5-HT. (**A**) Effect of 5-HT pretreatment on the 5-HT uptake ability of the endothelial cells. Endothelial cells in one well of a 24-well plate (2 × 10^5^) were pretreated with (0–300 μM) 5-HT for 45 min at room temperature before uptake rates of [^3^H]-5HT were measured in intact cells Rate measured over three independent experiments, (p < 0.001). (**B**) Effect of 5-HT pretreatment on the surface expression of SERT. Endothelial cells were pretreated with 0, 20, or 100 μM 5-HT and biotinylated with NHS-SS-biotin^16^,^20^,^22^. Biotinylated plasma membrane proteins were retrieved on streptavidin beads and analyzed for SERT by WB analysis. Intracellular SERT was determined by WB analysis of non-bound material. Cells without 5-HT pretreatment served as a control. Data are representative of at least three independent experiments. Actin served as a loading control. The results of WB analysis are the summaries of combined data from three densitometric scans (mean ± SD). *represents differences from 0 μM 5HT-matched samples (P < 0.001).

**Figure 4:** 5-HT-mediated phosphorylation of vimentin. (**A**) IF and (**B**) WB analysis of endothelial cells pretreated with 5-HT. Vimentin (green) and its phosphorylated form, P-vimentin (red) were visualized by confocal microscopy in control endothelial cells and in cells pretreated with 5-HT. DNA was stainind with DAPI. Note both character an the intensity of P-vimentin staining was changed in cells pretreated with 5-HT. The bar is 10 μM. Figures show representative images from at least 2 separate experiments. WB analysis of endothelial cells confirmed IF data showing the phosphorylation of vimentin following 5-HT pretreatment. (**C**) 5-HT signaling and P-vimentin formation. Platelets endogenously express vimentin (lanes 1–4)) and in the 5-HT pretreatment vimentin is phopsphorylated only in the platelets of WT mice (lane 2). However platelets of SERT KO mice did not permit the phosphorylation of vimentin (lane 4). These findings indicate the involvement of 5-HT signaling in P-vimentin formation in the platelet cytoplasm.

The article "Sepsis-induced elevation in plasma serotonin facilitates endothelial hyperpermeability" was retracted in 2019. Reasons: errors in the images; original data or images not available.

**Figure 5:** TGase and 5-HT in P-vimentin formation. (**A**) In exploring our hypothesis in the involvement of TGase in phosphorylation of vimentin, endothelial cells (2 × 10^5^ cells/assay) were treated with TGase inhibitor Cys and our experimental condition was PAR-treated endothelial cells. Endothelial cells were pretreated with 20 μM 5-HT or Cys or PAR or 5-HT + Cyst/PAR. The whole cell lysate were resolved on SDS-PAGE followed by WB analysis using a polyclonal P-vimentin or vimentin-Ab. Densitometric scanning of the immunoblots in was performed, and *asterisks* indicate samples that significantly differ between the groups. Results from three independent experiments are shown (mean ± S.D. (error bars)). While 5-HT pretreatment mediated the phosphorylation of vimentin (lane 2), the presence of Cys or PAR ceased the upregulatory role of 5-HT in P-vimentin formation (lanes 3 and 4). (**B**) PAK and P-vimentin formation and ve-cadherin association with P-vimentin. Endothelial cells (2 × 10^5^ cells/assay) were treated with 20 μM 5-HT or Cys or 10 μM PAR1 inhibitor, PAR1-18. Pretreated or control endothelial cells were lysed and a portion of it was saved for WB analysis with PAK1- or P-PAK1- or actin-Ab. The rest of the cell lysates were prepared for the co-IP assay with P-vimentin Ab (polyclonal) coated sepharose A beads. The IP were eluted and subjected to WB analysis with ve-cadherin Ab (monoclonal). The level of P-vimentin on was found elevated in 20 μM 5-HT pretreated cells; but this elevation was stored in PAR treatment. Nonspecific adsorption of Sepharose beads was not determined in the absence of vimentin-Ab. Figures show representative images from 3 separate experiments. Actin was used as a loading control. Quantification of the results from the panel was performed by densitometric scanning and presented after normalized with actin. The association between cadherin and P-vimentin was 4.25-fold higher in 5-HT pretreated, 1.86-fold higher in 5-HT and Cyst or PAK1-18 treated endothelial cells than the control group indicating that P-vimentin can be formed in different pathways although 5-HT signaling is the major one. This result is significantly different from the level of 5-HT + Csyt or 5-HT + PAR treated samples association (two-sided t test, p < 0.05). Results from three independent experiments are shown (mean ± SD).

The article "Sepsis-induced elevation in plasma serotonin facilitates endothelial hyperpermeability" was retracted in 2019. Reasons: errors in the images; original data or images not available.

**Figure 6:** RIP of ^3^H-5HT labeled Rac. Endothelial cells are treated with 20 mM 5-HT alone (lane 2) or 20 min after PAR (lane 3) or Cyst (lane 4) treatments. At the end of incubation time [^3^H]-5HT was included in PBS/CM at room temperature. After 1 hr, cells were washed with ice cold PBS and harvested. Samples from: (i) whole cell lysate; (ii) the proteins pulled down by Rac-Ab; and (iii) depleted cell lysates after Rac-Ab pull were normalized based on their protein concentration. Then, equal amount of samples from each group were mixed with 5 ml scintillation cocktail and measured in the scintillation counter (bar graph). Immune precipitates were eluted from the beads by incubation in SDS sample buffer, analyzed by 12.5% SDS-PAGE, and Rac was visualized by fluorography. A 25 kD major band representing Rac was precipitated with anti-Rac Ab only from the cells of 5-HT-treated. PAR- or Cyst-treatment inhibits the serotonylation of Rac. The whole cell expression of SERT and Rac were determined by WB of endothelial cells, which shows that PAR or Cyst treatment did not change the level of SERT or Rac. Data are representative of at least three independent experiments (mean ± SD).

**Figure 7:** Effects of 5-HT on extravasation of FITC-dextran from murine endothelial cells *in vitro*. Endothelial cells (2 × 10^5^ cells/assay) grown on Transwell-COL 24 mm diameter 0.04 μm pore size plates inserts were either treated with 5-HT or together PAR and 5-HT or proceed to the assay directly without treatment as control. FITC-dextran (40 kDa) was introduced into the upper compartment and the lower compartment was sampled after 45 min. 5-HT (20 μM) revealed a significant 1.32-fold increase in leakage in the absence of other serum factors. However, in the presence of PAR, 5-HT pretreatment was not effective. Data are mean ± SD, n = 10 replicates; *p < 0.05 compared to Control.

**Figure 8:** Role of SERT *in vivo*. Mice were made septic by CLP and microvascular leakage was assessed using Evans Blue dye at 4 h post-CLP (**A**) CLP produced a significant increase in kidney levels of Evans Blue dye, which was prevented by paroxetine (PAR, 4 mg/kg, ip) administered at the time of CLP (n = 4–5 mice/group). In separate experiments, renal cortical capillary perfusion was assessed using IVVM at 6 h post CLP (**B**) CLP produced a significant decline in perfusion, which was improved by PAR administered at the time of CLP. SERT^−/−^ mice also had improved perfusion (n = 4–6 mice/group). Representative still images from the captured videos are presented in panel (**C**). White arrows point to capillaries with no blood flow. Data are mean ± SE. *P < 0.05 compared to WT CLP and ^†^P < 0.05 compared to WT SHAM.

The article "Sepsis-induced elevation in plasma serotonin facilitates endothelial hyperpermeability" was retracted in 2019. Reasons: errors in the images; original data or images not available.

**Figure 9:** Proposed mechanism by which 5-HT signaling and SERT facilitates endothelial hyperpermeability during sepsis. The data suggest that during, sepsis increased levels of platelet-derived 5-HT initiate intracellular signaling pathways in the endothelial cell, through the activation of TGase and the phosphorylation of vimentin on Ser56^22^. Following phosphorylation, the curved filamentous structure of vimentin undergoes reorganization and straightens^14^,^15^. Ve-cadherin binds tightly to P-vimentin and induces a weakening of the cellular junction. This results in vascular microvascular leakage.
